# The Influence of Identity and Management Skills on Teachers' Well-Being: A Public Health Perspective

**DOI:** 10.1155/2022/3156133

**Published:** 2022-08-09

**Authors:** Huiqing Zhang

**Affiliations:** Faculty of Education, National University of Malaysia, Bandar Baru Bangi 43600, Malaysia

## Abstract

At present, the state and society pay more and more urgent attention to higher education, and higher education has transitioned from elite education to mass education. College teachers, as the main force in the construction and development of colleges and universities, have the right to pursue professional happiness. Their professional happiness is not only related to themselves but also related to the growth of college students and the development of higher education. Therefore, this paper deeply studies the connotation of teachers' professional happiness, analyzes the current situation of their professional happiness, the current happiness level of college teachers, and discusses the strategy of improving college teachers' professional happiness, which has great value and significance to the development of national higher education.

## 1. Introduction

University professors who have a sense of well-being are more passionate about their university teaching profession and are better able to teach professional knowledge, while they can spread more positive energy and convey the right outlook to university students, laying a good moral foundation for them to enter society. So university professors, as a public profession, influence the moral and intellectual well-being of the future mainstay of society, and their well-being is a public health issue. This paper is, therefore, appropriate for this journal.

Nowadays, the state and society are paying more and more urgent attention to the quality of education. The report of the 18^th^ National Congress of the Communist Party of China emphasized that education is the cornerstone of national rejuvenation and social progress. As an important part of education, higher education has transitioned from elite education to mass education and has trained and delivered a large number of high-quality talents to the country[1]. College teachers are the main body of college development and the first resource of education. Only with the backing of outstanding college teachers can colleges and universities achieve stable development. Whether college teachers can devote themselves to teaching with a full and enthusiastic attitude largely depends on their professional well-being. If teachers do not have high professional happiness, there will be no high-quality work with an innovative and selfless spirit, which will also directly affect the quality of higher education.

On August 11, 2014, Tencent Education launched a survey on the living conditions of teachers. It collected nearly 420,000 questionnaires from teachers in schools through online surveys and surveys without sampling and testing in an attempt to show the current living conditions of teachers. Overall, more than 80% of teachers said that the work is heavy, reflecting the high pressure of work. Nearly 30% of teachers are in poor health and are in a state of fatigue. More than 90% of teachers are dissatisfied with their actual wages. About 40% of teachers' wages have not risen in three years, and nearly 70% of Cheng teachers believe that society does not respect the teaching profession, and nearly 50% of teachers say they will never let their children take up the teaching profession. Such survey results reveal that the current pressure, income, and social status of teachers in my country are not optimistic, and it is very difficult for the majority of teachers to perceive happiness in their occupations [2].

In recent years, research on teachers' professional well-being has gradually become a hot topic. Paying attention to the professional well-being of teachers in colleges and universities and exploring the attributions that affect teachers' professional well-being are of positive significance for improving teachers' management policies, ensuring teachers' physical and mental health, maintaining teachers' sustainable development, and stabilizing the teaching staff. Through the analysis of the research fields, it can be seen that most of the current research focuses on the occupational well-being of teachers in primary and secondary schools, while the research on the occupational well-being of teachers in colleges and universities is still insufficient. Therefore, this paper focuses on the impact of identity and management skills on teachers' well-being [1, 3–5]. Through the interview and survey of the occupational health status of university teachers, the current happiness level of university teachers is understood, and the corresponding research strategies are proposed based on the research results, which is of great value and significance to the development of national higher education.

## 2. State of the Art

### 2.1. Happiness

Well-being is the science of good human existence. The study of well-being in the field of psychology began in the 1990s and 1990s, represented by Western countries. The research on well-being stems from the birth of a new school, positive psychology, advocated by the psychology community [6]. Positive psychologists believe that happiness is the most basic emotional need of everyone. The World Federation of Mental Health also includes the standard of happiness as one of the four standards of mental health. There are also different schools of view on happiness in my country. Among them, the schools of certain representative significance include Confucianism, Taoism, and Buddhism as shown in Table 1

In his writings, Marx expounded the Marxist concept of happiness, believing that if people can choose the labor occupation that can best benefit mankind and contribute to the development of mankind, then difficulties and setbacks will not knock people down because that kind of happiness belongs to the masses, all those who are helped, not selfish, limited, and noble people will shed hot tears in the face of the ashes of those who are dedicated. From the interpretation of this classic concept of happiness, it can be seen that the people-oriented concept of Marx's concept of happiness is the theoretical basis, collectivism is the ultimate goal, and overall consideration is the fundamental method [7].

The theory of happiness is used to study the happiness level of college teachers so as to understand the mental health problems of college teachers. With the people-oriented world theme and the continuous advancement of my country's quality education, my country's education has gradually entered an era of focusing on student development. For a long time, the focus of research in the education sector has been mainly on the development of teachers' professionalism in order to further standardize the teaching staff, to better serve society and students, ignore the concern for teachers' spiritual life, and lack humanistic care for teachers' pursuit of a happy life. However, in recent years, the academic community has gradually realized the consequences of this neglect, and the quality of life of teachers, especially the problem of teachers' well-being, has increasingly come into people's perspective [8]. At present, the definition of teachers' well-being can be roughly divided into three categories: one is the concept of subjective well-being, which is based on the philosophy of “happiness theory,” which refers to an individual's overall evaluation of his life according to his own standards and emotional experience. Its operational indicators include life satisfaction, positive affect, and negative affect. Xiao Jie's definition of teachers' well-being falls into this category. He proposes that teachers' professional well-being is the continuous and stable happy experience of teachers' work based on their own standards. Another category adopts the concept of psychological well-being, and its philosophical background is “realization theory.” Psychological well-being emphasizes the full realization of people's potential and emphasizes people's positive self-esteem, social service, the purpose of life, and the universal significance of friendly relationships, which constitute the core elements of psychological well-being [9].

In this paper, happiness is defined as the personal satisfaction obtained by people in the social practice of creating living conditions due to the realization of personal, collective, and even human goals, ideals and justice, and public welfare. Happiness is the warm flow of passion between people from the heart to the deep sea of love; it is the simplicity of kind people. When people pay the sweat of responsibility, their foreheads must emit the light of happiness. In short, happiness is the feeling that people's desires are satisfied or partially satisfied, a kind of spiritual pleasure. Happiness is a subjective feeling of life satisfaction.

Teachers' professional well-being is produced by individuals engaged in educational and teaching activities and obtained after realizing their own values and exerting their own strengths experience. It is not only an important content of teachers' professional life but also an important criterion for evaluating the quality of their work and life [10]. Because happiness comes from identity, and teachers' happiness comes on the one hand from students' identification of their work, and on the other hand, comes from the social identity of their own identity.

### 2.2. Identity

Identity phenomena are very common in social life, such as social identity, cultural identity, national identity, national identity, and political identity. “Identify” has two meanings in modern Chinese: one is to feel kindly because of the common ground with oneself, and the other is to admit and recognize. At present, we can divide the interpretation of identification into two categories. The first category is to equate identification with “self-identification,” that is, an emotional driving force for individuals to establish connections with others and a need to seek psychological safety. The second category of explanations, such as James, Freud, Zhu Zhixian, Liang Liping, etc., equates identification with “the establishment process and result of self-concept,” that is, the process of individual personality self-formation, which refers to the moral field of adolescents or children. Psychological adaptation mechanism [11]. As explained in the American Psychological Encyclopedia, teachers' professional identity is teachers' awareness, emotion, expectation, will, values, and perception of their own professional skills. Teachers' professional identity is both a process and a state. As a “process,” a teacher's professional identity is the process in which the individual self gradually develops from his own experience and confirms his role as a teacher.

### 2.3. Management Skills

Teacher education management ability refers to a kind of behavior performance in the management process established and maintained by teachers in order to achieve the teaching objectives. The level of teachers' educational management ability directly affects the quality of teachers' teaching and also greatly promotes or negatively affects students' learning. Teachers are the main force in curriculum reform and the key to basic education curriculum reform, and teachers' educational management ability is an important guarantee for teachers' effective teaching [12, 13]. As a teacher not only must master the relevant professional knowledge and professional skills but must also have certain appropriate teaching abilities only in order to carry out effective classroom teaching, to ensure the smooth realization of educational and teaching goals, to comprehensively improve the quality of teaching, and strive to cultivate qualified talents for building a harmonious society. Classroom teaching ability is a direct and effective tool and means to complete teaching tasks, and it is the concentrated expression of teachers' education and teaching ability. This is not only related to the overall improvement of the quality of education and enrollment but also directly related to the development of students' thinking ability. It can be said that classroom teaching ability is the basic ability that teachers must possess, an important part of teachers' professional ability, and also directly affects the classroom. The efficiency of teaching activities improves the classroom teaching ability to successfully complete the classroom teaching activities.

### 2.4. Influencing Factors of Teachers' Well-Being

Scholars at home and abroad have conducted relevant research on the influencing factors of teachers' well-being from various aspects, and the research results are basically consistent. According to the research, the influencing factors of teachers' well-being can be roughly divided into the following categories: Demographic variables include age, gender, school type, marital status, professional title, etc. The results of a survey on the occupational well-being of Dutch teachers show that the elderly teachers have a very high level of well-being. Teaching subjects and teachers' own level will cause the biggest difference in teachers' occupational well-being. Teachers in vocational schools have the lowest level of well-being. The ones who are teachers of special courses in comprehensive middle schools. The study found that the relationship between job satisfaction and age, which is a measure of job well-being, is in the form of a *U*-shaped curve. The results of the domestic questionnaire survey on the subjective well-being of primary school teachers show that there are significant differences in the subjective well-being of the genders, male teachers' well-being is higher than that of female teachers. Yang Wanqiu's research on the subjective well-being of primary and secondary school teachers found that there are significant differences in the subjective well-being of primary and secondary school teachers in terms of regional factors where teachers come from. Cao Guanghai's research on the subjective well-being of higher vocational teachers found that higher vocational teachers of different genders, ages, professional titles, and marital profiles, while this paper mainly explores the happiness level of college teachers from the two factors of identity and management skill level.

## 3. Interview Survey on the Current Situation of Professional Well-Being of College Teachers

### 3.1. Basic Situation

In order to gain an in-depth understanding of the current status of teachers' professional well-being in a certain college and then explore the reasons for the happiness and unhappiness of college teachers, and seek strategic help for the improvement of teachers' happiness, this study selects 300 teachers from a college with different backgrounds and uses the following methods. The interview method combines quantitative research with qualitative research to jointly study teachers' professional well-being in order to provide a qualitative research basis for the questionnaire survey and improve the authenticity of this paper. The basic information of teachers is shown in Table 2 and Figure 1:

After sorting out and analyzing the salary part of teachers' happiness satisfaction in the survey data obtained, relevant conclusions can be drawn. The salary level of teachers is unevenly distributed, and the number of people in the four grades is different. Only 46% of teachers are relatively unsatisfied with the current salary level. Satisfied, the specific data is shown in Figures 2 and 3.

### 3.2. Happiness Survey

According to the teachers' targeted survey and statistics on the happiness of each part of the teaching and work, survey and research on various aspects of happiness, and explore happiness from multiple dimensions, as shown in Table 3:

After sorting it into a chart, it is found that teachers' happiness in terms of the working environment and salary treatment is significantly lower than in other aspects, and there is a lot of room for improvement. This is mainly because the salary level of college teachers is relatively not high, the working environment is affected by the level of universities, and there are certain differences, resulting in the following results. See Figure 4 for details.

Moreover, teachers of different genders also have great differences in happiness. It can be seen that the happiness index of female teachers is higher than that of male teachers, and the happiness rate is higher, as shown in Figure 5:

In order to understand whether there are differences in the well-being of teachers of different genders, an independent sample test was used to conduct variance analysis. The test results are shown in Table 4.

As can be seen from Table 4, the happiness index of teachers of various genders is generally at the upper middle level (total score is 7), but there are significant differences in the level of happiness of teachers of different genders. Among them, the happiness index of female teachers is 5.61, which is higher than the male happiness index of 5.03, mainly because the social pressure on men is greater than that on women.

## 4. Result Analysis and Discussion

After analyzing the survey results, it is found that the overall subjective well-being level of college teachers is at a high level, which may be related to the professional characteristics of college teachers: college teachers are a special group responsible for teaching, scientific research, administrative management, and service. Teachers who are competent for this position are selected from outstanding applicants, with high comprehensive quality in all aspects, and the age of the teaching team is gradually showing a younger trend, able to actively and effectively deal with pressure and resolve negative emotions. In all dimensions of happiness, the respondents showed higher scores, which may be related to the living environment and work characteristics of college teachers. The friendly and altruistic working environment of college teachers, whether it is teaching and scientific research or management and service work, requires strong group collaboration. In a good working atmosphere, self-worth and health and vitality are more likely to be improved. The two are a virtuous circle of mutual promotion, which can jointly improve the well-being of college teachers.

The professional identity of college teachers is highly correlated with teachers' happiness. The specific rule is that the higher the degree of teachers' professional identity, the higher the level of happiness, and the specific experimental results are shown in Table 4. At present, there are few domestic studies on the relationship between the two. Yu Songhua and others have done a related study on teachers' professional identity and happiness index and found that teachers' professional identity and its factors are significantly positively correlated with teachers' happiness index. The research results are basically the same. Teacher teaching is the most important job for teachers, and teaching is a way for teachers to achieve personality growth and obtain positive emotions. When teachers cannot agree with this job, it means that teachers cannot accept it. The self in the teaching process cannot be developed freely in teaching, nor can one experience positive emotions such as joy, happiness, and pride in teaching, and the idea of resignation arises spontaneously. It can be seen that personality growth and positive emotions are the most direct factors in the process of resignation intention, while occupational identity indirectly affects resignation intention due to its great influence on personality growth and positive emotions [14–17].

The improvement of teachers' management skills will improve teachers' classroom comfort, teachers' classroom atmosphere is good, and students' interest in learning is high so that both parties can experience happiness in the process of education, teaching, and learning, and teachers' happiness will also be improved accordingly. Therefore, improving teachers' management skills is of great significance to improve teachers' well-being.

## 5. Suggestions for Improving the Well-Being of College Teachers

### 5.1. Create a Humanized Campus Atmosphere and Create Harmonious Interpersonal Relationships

Social attributes are the basic attributes of people, and society has a huge impact on people, including not only personal development but also happiness. Colleges and universities are small societies where teachers work and live. Teachers' interpersonal relationships are mainly divided into leadership relationships, teacher-student relationships, and family relationships. These relationships have an important impact on teachers' subjective well-being. As university leaders, we can effectively improve teachers' subjective well-being around these aspects. School leaders and all teachers should work together to create harmonious interpersonal relationships and build a people-oriented campus atmosphere. First of all, the leadership team of the school must reach a consensus, set an example first, form spiritual cohesion, and take overall consideration when distributing honors and awards, so as to enhance the harmony of interpersonal relationships between faculty and staff; it is necessary to promptly resolve any unhealthy trends that may exist among teachers. It is necessary to stop it in a timely manner and criticize some teachers in a timely manner when they need to be criticized; at the same time, it is necessary to create cooperation opportunities among teachers, weaken competition, relieve teachers' professional pressure, and help teachers work and live happily. Secondly, teachers should pay attention to communication with colleagues and students. Schools can create a platform for teachers to communicate with each other. Through communication, teachers can strengthen cooperation and friendship, resolve existing misunderstandings in a timely manner, and build harmonious relationships with colleagues; communication can timely understand students' learning and psychological conditions, make their teaching content more targeted, and can also form an atmosphere of mutual understanding and mutual support between teachers and students, and create a harmonious teacher-student relationship [18].

Colleges and universities should not only promote the healthy growth of students by creating a good and positive school spirit and study style, but also encourage teachers to devote themselves to their work by creating a vibrant and harmonious educational and teaching atmosphere. Therefore, colleges and universities should fully respect and understand the reasonable needs of teachers and provide more training and further study opportunities while helping them solve their difficulties in life so as to help them better realize their own development and adapt to education, teaching, and subject professional development. It should build a platform for promoting teachers' self-development and self-value. While encouraging teachers to put forward reasonable demands that are conducive to education, teaching, and scientific research, they should strictly urge relevant departments of the school to assume the responsibility of serving teachers.

### 5.2. Improve Teachers' Salary Level and Academic Reward Level

Colleges and universities should establish a “people-oriented” management concept, create a teacher performance assessment system based on the different requirements for teachers at different levels, and adopt a variety of assessment methods to conduct targeted assessments on teachers' teaching and scientific research; at the same time, follow the teaching work of higher education. Guided by modern human resource management theory, the transparency of teachers' performance assessment and evaluation will be further improved so as to make a more objective and fair evaluation of teachers' work performance.

The work level of personnel managers in colleges and universities directly affects the quality of personnel work in colleges and universities. In order to formulate a scientific and standardized management system and implement it smoothly, personnel management workers in colleges and universities need to have solid management professional knowledge and skilled professional skills, as well as master advanced management methods; they also need to accumulate rich humanities and social sciences. Knowledge, uphold justice, abide by professional ethics and guidelines, and be good at communicating and communicating with teachers on an equal footing [19]. Therefore, colleges and universities should actively create opportunities for vocational training for personnel management workers, not only focusing on the training and improvement of their professional ability but also on the training and improvement of their professional ethics and interpersonal skills so as to facilitate the smooth operation of personnel management in colleges and universities and lay a good foundation for development.

Although material conditions cannot directly determine an individual's subjective well-being, it is an indispensable and important factor. In the interview, it was also found that the salary of college teachers is not equal to their work, and many teachers hope to improve their salary. Therefore, the competent education department should comprehensively consider the social and economic level and price level, adjust teachers' salaries in a timely manner, improve teachers' living standards, and relieve teachers' worries about their work. In addition, interviews with teachers with different professional titles also found that professional titles have a greater impact on teachers. Many teachers hope to improve their scientific research ability through training opportunities and reward mechanisms. Therefore, schools can consider providing teachers with more scientific research exchanges and cooperation, provide teachers with better scientific research resources, set up a reasonable scientific research assessment mechanism, increase the reward mechanism, and enhance the enthusiasm of teachers in scientific research, thereby improving teachers' scientific research ability and allowing more teachers to experience higher levels in the process of self-realization and subjective well-being.

### 5.3. Pay Attention to the Well-Being of Young Teachers in Colleges and Universities

For young teachers in colleges and universities, although they have a relatively high social status among their peers, their economic income level is not equal to it. There has been a study that the overall income of college teachers belongs to the upper middle level, but the phenomenon of polarization is more obvious: the income level of college teachers with high positions, high professional titles, and scientific research backbones is higher, while the income of young teachers is often low. Young teachers also need to bear high-intensity work pressure, housing prices, and various family pressures, so their subjective well-being is not optimistic. For the new young teachers in colleges and universities, they have to bear all kinds of pressure. For colleges and universities, they should attach great importance to the work and life status of young teachers, and create a reasonable promotion channel, excellent resource support, and harmonious interpersonal atmosphere for them, a fair evaluation system, and at the same time, pay attention to the difficulties in their lives and solve them in time, so as to alleviate the “worries” of young teachers so that they can work in a good mental state to make greater contributions [20].

In addition to spending a lot of time with students, teachers spend the rest of their working time basically spending time with colleagues. Maintaining a good relationship with colleagues is an important foundation for teachers to carry out their work. Therefore, colleges and universities should vigorously advocate sincere treatment among colleagues and maintain a good cooperative attitude and guide teachers to form a humble and prudent way of doing things and an enthusiastic and open positive attitude, so that teachers can appreciate the advantages of colleagues and correct their own shortcomings. When problems arise, they can deal with them calmly and peacefully and can ensure smooth communication among colleagues with good communication methods so that teachers can gain comfort and happiness in their interactions with colleagues.

### 5.4. Establish Teachers' Professional Well-Being

Teachers have always been considered the most sacred profession in the world. What they face every day is not machines that cannot speak but many young, energetic, and promising young people. Teachers' work includes a lot of interaction between teachers and students, and teachers' words and deeds influence students in various ways. When students finish their studies, leave the campus, go to work, and contribute to national development and social progress, “Education of the world's talents,” at this time teachers' sense of achievement and happiness is the highest.

Colleges and universities can establish an active support system by establishing a teacher's physical and mental health evaluation system and regularly collect, analyze, process, store, extract, and evaluate teachers' relevant information. Through this active support system, active support is provided to teachers with problems in the early stage of teachers' physical and mental health assessment to avoid the deterioration of the situation; at the same time, for teachers with problems, it is further confirmed whether they are in a state of crisis through psychological examination; Teachers who are confirmed to be in crisis will be provided active support services by relevant school departments through psychological counseling or workshops.

### 5.5. Reasonably Release Pressure

In the face of heavy education, teaching, and research tasks, as well as the objective pressure of interpersonal communication with students, colleagues, and school leaders at all levels, teachers will have a greater ideological burden in their professional behavior. Therefore, for colleges and universities, it is imperative to build an efficient communication platform for two-way interaction between front-line teachers and school administrators. A good relationship between superiors and subordinates can help reduce teachers' interpersonal pressure. The open and two-way interactive communication channel is not only an effective way for school managers to directly understand the demands of front-line teachers, but also an effective way for teachers to release work pressure. Through a two-way interactive and efficient communication platform, on the one hand, school administrators can keep abreast of teachers' teaching environment so as to eliminate unfavorable factors affecting their professional behavior as much as possible for teachers; on the other hand, teachers can timely understand and grasp the implementation of school administrators It lays a good foundation for the efficient realization of educational and teaching goals.

As contemporary, in addition to enjoying the convenience and comfort of various modern technologies, we are also bearing various life pressures, social responsibilities, and family burdens. Individuals who are under multiple pressures need to expand their stress relief channels and learn to seek help in a timely manner for those who need help in the workplace or in the collective; at the same time, family and friends are an important part of individual stress relief and social support. A person with a good social support system, even if he encounters setbacks or failures, will turn adversity into prosperity, from misfortune to happiness. In addition to the benign support from the external environment, individuals should also find more reasons for themselves, set reasonable goals, and choose work content in a targeted manner. Enhance your ability to deal with stress and confusion. As a college teacher, in fact, the characteristics of work have more advantages than ordinary people, and teachers often have more free time for their own disposal. It is a good way to learn to use this time reasonably and effectively. You can choose appropriate exercise methods to regulate your body and mind, and you can use this time to improve and optimize your social support system so as to maintain a good physical and mental state, enhance your ability to cope with stress, and gain higher happiness experience. No matter what kind of work pressure is faced, teachers should treat their work with a positive and optimistic attitude, and at the same time, should also have more brave perseverance and courage. The domestic society has always been biased towards education and may not necessarily hold a positive attitude towards the teaching profession. This social reality has a negative impact on the professional identity of college teachers. Teachers should accept the reality, abandon the prejudice against school students, teach hard, and prove the value of the teaching profession with their own practice. When teachers encounter difficulties in work and life, they can accept help from the school or others, but more fundamentally, they should face problems with optimism and open-mindedness and learn to relieve various negative emotions by themselves.

### 5.6. Improve the Identity of Teachers

Pay attention to planning, meet the needs of teachers' occupational safety, and enhance teachers' professional identity. Colleges and universities should clearly recognize that an excellent team of teachers has a guarantee of teaching quality, which is also the core driving force of school development. Therefore, “doing a good job in human resource planning, improving teachers' treatment, and reducing the loss of excellent teachers” should be a key work of colleges and universities. Due to the low antirisk ability and unclear development goals of colleges and universities, also because the teacher is a career that needs to progress with time, the level of personal ability will also cause teachers to have a low sense of occupational security. Therefore, the organizers of colleges and universities should make long-term plans for the development of the school, clarify the development path of the school, and strive for the long-term and stable development of the school. Only in this way can a solid career development platform meet the “safety needs” of teachers, enhance their sense of occupational security, and cultivate their sense of belonging to the school, which has a positive effect on promoting the stability of the teaching staff in colleges and universities.

## 6. Conclusion

In the current environment of paying more and more attention to higher education, the happiness level of college teachers directly determines the work quality of college education.

This paper deeply studied the connotation of teachers' professional happiness, analyzed the status quo of teachers' professional happiness and the current happiness level of college teachers, and found that college teachers have lower happiness in salary and working environment, and the happiness index of women is higher than that of men. Based on the above research conclusions, the paper also discusses the specific strategies for improving college teachers' professional happiness, which is of great value and significance to the development of national higher education.

## Figures and Tables

**Figure 1:** Teachers' teaching age.

**Figure 2:** Teacher salary levels.

**Figure 3:** Teachers' salary satisfaction.

**Figure 4:** The happiness index in different aspects.

**Figure 5:** The happiness index of different genders.

**Table 1:** Different schools of thought on happiness.

Representative school	The main point of happiness
Confucianism	Advocating morality as the root of all things, happiness is no exception. Take virtue as happiness and happiness as the thought of happiness, and everything is good.
Taoism	It is advocated that everything should be natural, not to be forced, to be pure of heart and few desires, to look at everything in a plain way, to be happy, and to be one with happiness naturally.
Buddhist	It is advocated that letting nature take its course, happiness comes from the heart, and whether happiness is a subjective idea of oneself. Looking at the world plainly, calming down your mind, and properly controlling your mind will bring you happiness.

**Table 2:** Basic information of teachers.

	Basic situation	Number of people (people)	Proportion (%)
Gender	Female	226	75.3
	Male	74	24.7

Age	30∼33 years old	21	7.0
	34∼36 years old	79	26.3
	37∼40 years old	106	35.3
	41∼44 years old	74	24.7
	45∼48 years old	20	6.7

**Table 3:** Meanings of various aspects of happiness.

Module	Dimension	High scorers explained
Subjective well-being	Life satisfaction	The individual's needs and desires are met in all aspects, and the individual is satisfied with his or her life situation
	Positive emotions	More time to experience positive emotions such as love, joy, happiness, pride, optimism, etc.
	Negative emotions	Experience more negative emotions such as depression, anxiety, jealousy, anger, guilt, etc.

Psychological well-being	Vitality	Full of energy, feeling of energy, with a passion for life, full of energy
	Health concern	Cherish life, pay attention to health, maintain a good way of life and behavior
	Altruistic	Be willing to help others, be caring, and hope to make the world a better place through their own efforts
	Self-worth	Believing in one's own abilities and importance, having a sense of accomplishment and worth, and having high self-esteem
	Friendly	Relationships have warm, safe, genuine, lasting relationships
	Personality	Growth, self-acceptance, continuous development, openness to new experiences, self-awareness, ability to control one's own behavior
Happiness index		Feeling very happy throughout life	

**Table 4:** Differences in subjective well-being of teachers of different genders.

Gender	*M*	*T*	*P*
Male	5.03	−3.265	0.002^*∗∗*^
Female	5.61		

## Data Availability

The labeled data set used to support the findings of this study is available from the author upon request.
